The article "Tanshinone IIA Induces Apoptosis in Human Oral Cancer KB Cells through a Mitochondria-Dependent Pathway" was retracted in 2017. Reasons: contaminated cell lines or tissues; unreliable results or conclusions.

# Tanshinone IIA Induces Apoptosis in Human Oral Cancer KB Cells through a Mitochondria-Dependent Pathway

**DOI:** 10.1155/2014/540516

**Published:** 2014-05-13

**Authors:** Pao-Yu Tseng, Wei-Cheng Lu, Ming-Ju Hsieh, Su-Yu Chien, Mu-Kuan Chen

**Affiliations:** ^1^Department of Otorhinolaryngology, Head and Neck Surgery, Changhua Christian Hospital, No. 135 Nanxiao Street, Changhua 500, Taiwan; ^2^Cancer Research Center, Changhua Christian Hospital, Changhua 500, Taiwan; ^3^Institute of Medicine, Chung Shan Medical University, Taichung 500, Taiwan; ^4^School of Optometry, Chung Shan Medical University, Taichung 402, Taiwan; ^5^Department of Pharmacy, Changhua Christian Hospital, No. 135 Nanxiao Street, Changhua 500, Taiwan; ^6^School of Pharmacy, China Medical University, Taichung 404, Taiwan; ^7^College of Health Sciences, Chang Jung Christian University, Tainan 711, Taiwan

## Abstract

Tanshinone IIA (Tan IIA), an active phytochemical in the dried root of *Salvia miltiorrhiza* Bunge, has shown an antiproliferative activity on various human cancer cell lines including nasopharyngeal carcinoma cells. However, the effects of Tan IIA on human oral cancer cells are still unknown. This study aimed to investigate the antiproliferative effects of Tan IIA on human oral cancer KB cells and explored the possible underlying mechanism. Treatment of KB cells with Tan IIA suppressed cell proliferation/viability and induced cell death in a dose-dependent manner through sulforhodamine B colorimetric assay. Observation of cell morphology revealed the involvement of apoptosis in the Tan IIA-induced growth inhibition on KB cells. Cell cycle analysis showed a cell cycle arrest in G_2_/M phase on Tan IIA-treated cells. The dissipation of mitochondrial membrane potential observed by flow cytometry and the expression of activated caspases with the cleaved poly (ADP-ribose) polymerase under immunoblotting analysis indicated that Tan IIA-induced apoptosis in KB cells was mediated through the mitochondria-dependent caspase pathway. These observations suggested that Tan IIA could be a potential anticancer agent for oral cancer.

## 1. Introduction

The incidence of oral cancer increases annually with the epidemiology of oral and oropharyngeal cancer, grouped together, as the sixth most common cancer worldwide [1]. It is estimated that about 275000~300000 people will be diagnosed with oral cancer annually [1, 2]. The management of oral cancer is complex and challenging. The majority of treatment includes surgery alone for very early stage patient, surgery with adjuvant concurrent chemoradiotherapy or radiotherapy alone, neoadjuvant chemotherapy followed by surgery and adjuvant concurrent chemoradiotherapy in locally advanced disease, and chemoradiotherapy alone in certain status like inoperative cases [3–8].

The article "Tanshinone IIA Induces Apoptosis in Human Oral Cancer KB Cells through a Mitochondria-Dependent Pathway" was retracted in 2017. Reasons: contaminated cell lines or tissues; unreliable results or conclusions.

With many choices of treatment available, the role of chemotherapy is moving toward a more prominent position. The compounds extracted from the natural sources have been introduced into the chemotherapy of head and neck cancers. Taxanes including paclitaxel, the ingredient in the Pacific yew tree, and docetaxel, an extract of European yew tree, are cytotoxic agents that interfere with the microtubule structure and cause the pause of cell division [9, 10]. Paclitaxel and docetaxel have been used as chemotherapy agents to treat squamous cell carcinoma of the head and neck in selected patients with survival benefits in clinical practice [11–13].

Danshen, the dried root of* Salvia miltiorrhiza *Bunge, has been used for the treatment of coronary artery diseases and cerebrovascular diseases in traditional Chinese medicine. Tanshinone IIA (Tan IIA), a diterpene quinonic compound from the extractable ingredient of Danshen, has shown its ability to protect from H_2_O_2_-induced cell death in cardiac myocytes and macrophage [14, 15]. In addition, Tan IIA was reported to have the growth inhibitory effects and induced apoptosis on various cancer cell lines [16–19]. These studies indicated that Tan IIA could induce cell death through activation of selective members in caspase family and trigger the mitotic arrested cells to enter apoptosis [16, 17]. Yang et al. also pointed out that Tan IIA caused the release of cytochrome c, the loss of mitochondrial membrane potential, and subsequently the apoptosis of the EAhy926 human endothelial cells [19]. However, the effects of Tan IIA on human oral cancer cells are still unclear. This study was designed to investigate the cytotoxic effects of Tan IIA on human KB cells and discussed the possible underlying mechanism. Our data showed that Tan IIA may have the potential to become a novel agent of chemotherapy for oral cancer.

## 2. Materials and Methods

### 2.1. Reagents

Tanshinone IIA (Tan IIA) was purchased from Herbasin Co., Ltd. (Shenyang, China) and dissolved in pure grade dimethyl sulfoxide (DMSO). Dulbecco's modified Eagle's medium (DMEM), fetal bovine serum, penicillin, streptomycin, and 3, 3′-dihexyloxacarbocyanine iodide (DiOC_6_) were purchased from Gibco/Invitrogen (Carlsbad, CA, USA). The protein assay kit was obtained from Bio-Rad (Hercules, CA, USA). Antibodies to caspase-3, caspase-9, poly-(ADP-ribose) polymerase (PARP), and *β*-actin were purchased from Cell Signaling Technology, Inc. (Beverley, MA). PVDF membrane and chemiluminescent substrates for horseradish peroxidase (HRP) were purchased from Millipore (Bedford, MA, USA). Unless otherwise indicated, all other chemicals employed in this study were purchased from Sigma Chemical Co. (St. Louis, MO, USA).

The article "Tanshinone IIA Induces Apoptosis in Human Oral Cancer KB Cells through a Mitochondria-Dependent Pathway" was retracted in 2017. Reasons: contaminated cell lines or tissues; unreliable results or conclusions.

### 2.2. Cell Culture

The human oral squamous carcinoma KB cells were from ATCC (Manassas, VA, USA). The cells were cultured in DMEM supplemented with 10% fetal bovine serum, 100 units/mL penicillin, and 100 *μ*g/mL streptomycin at 37°C in one atmosphere with 5% CO_2_.

### 2.3. Cytotoxicity Assay

KB cells (8 × 10^3^ cells/well) were seeded in 96-well plate and grew overnight. Various concentrations of Tan IIA (0, 5, 10, 20 and 25 *μ*g/mL) were added and incubated for 24, 48, and 72 hours. The cell viability was determined by sulforhodamine B (SRB) colorimetric assay at different time periods.

For SRB colorimetric assay, 10%  wt/vol trichloroacetic acid was added to each well and the cells were then washed by tap water after 60 minutes. After dehydration, the plates were incubated in 0.4% SRB and then washed by 1% acetic acid after 15 minutes. Subsequently, 10 mM Tris buffer (pH 10.5) was added to dissolve precipitates. Finally, the optical density at 492 nm was measured to determine the cell viability.

### 2.4. Determination of Apoptosis and Morphologic Changes

KB cells treated with different concentrations of Tan IIA (0, 5, 10, and 20 *μ*g/mL) were incubated. At indicated time points (24 and 48 hours), the cells were fixed with 4% paraformaldehyde for 15 minutes at room temperature and kept incubating overnight at 4°C. Then, the plates were washed twice with phosphate-buffered saline (PBS) and nuclei were stained with 100 ng/mL Hoechst for 15 minutes in the dark. Following three times of tap water washing, the cells were examined under a fluorescence microscope. Cells with rough surface and dark stained nuclei with fragmented chromosome were considered as apoptotic cells. The apoptotic cells were counted for each sample.

### 2.5. DNA Cell Cycle Analysis

For the cell cycle analysis, the cellular DNA content was detected by flow cytometry. KB cells were plated in 6-well plates and incubated with Tan IIA (0, 5, and 10 *μ*g/mL) for 24 and 48 hours. The cells were harvested by centrifugation, washed with PBS, and fixed in 70% ethanol at −20°C overnight. Then, the cells were washed twice by ice-cold PBS and incubated in PBS containing 4 *μ*g/mL of propidium iodide, 0.1 mg/mL RNase A, and 0.1% Triton X-100 at room temperature for 1 hour in the dark. Finally, the cell cycle was analyzed with flow cytometry (Beckman FC500, San Diego, CA, USA).

### 2.6. Measurement of Mitochondrial Membrane Potential

KB cells were plated in 12-well plates and treated with different concentrations of Tan IIA (0, 5, and 10 *μ*g/mL) for 24 hours. The harvested cells were washed twice with PBS, resuspended in 10 *μ*M of 3,3′-dihexyloxacarbocyanine iodide (DiOC_6_), and incubated at 37°C for 30 minutes. Subsequently, the cells were analyzed with flow cytometry (Beckman FC500, San Diego, CA, USA).

The article "Tanshinone IIA Induces Apoptosis in Human Oral Cancer KB Cells through a Mitochondria-Dependent Pathway" was retracted in 2017. Reasons: contaminated cell lines or tissues; unreliable results or conclusions.

### 2.7. Western Blot Analysis for PARP and Caspase Activity

After incubation with Tanshinone IIA (0, 5, 10 and 20 *μ*g/mL) for 24 hours, KB cells were harvested and washed with cold PBS. Then, cell pellets were lysed in ice-cold RIPA buffer containing 20 mM Tris-HCl (pH 7.5), 150 mM NaCl, 1 mM Na_2_ EDTA, 1 mM EGTA, 1% NP-40, 1% sodium deoxycholate, 2.5 mM sodium pyrophosphate, 1 mM *β*-glycerophosphate, 1 mM Na_3_VO_4_, and 1 *μ*g/mL leupeptin for 5 minutes. The supernatants were collected by centrifugation at 11,752 g for 10 minutes at 4°C. The protein concentration was measured using the Bradford protein assay (Bio-Rad, Hercules, CA, USA). Proteins were electrophoretically separated on 8% sodium dodecyl sulfate-polyacrylamide gel electrophoresis (SDS-PAGE) gels and transferred to PVDF membrane. Membranes were supplemented with 5% nonfat dry milk and PBS containing 0.1% Tween-20 at room temperature for 1 hour. Then, membranes were incubated with diluted primary antibody against caspase-3, caspase-9, PARP, and *β*-actin at 4°C with gentle shaking overnight. After washing with PBST for three times, membranes were incubated with the appropriate horseradish peroxidase-conjugated secondary antibody at room temperature for 1 hour. Rewashing with PBST for three times, the blots were visualized using chemiluminescent detection reagents and autoradiographic film (Eastman Kodak Co., Rochester, NY, USA).

### 2.8. Statistical Analysis

Data were presented as the mean ± standard deviation (SD). Student's* t*-test was used for comparison among different groups. *P* < 0.05 was considered as statistically significant.

## 3. Results

### 3.1. Tanshinone IIA Inhibited Cell Growth and Caused Apoptosis of Oral KB Cells

To examine the cytotoxicity of Tan IIA on KB cells, the cells were evaluated by SRB colorimetric assay. The dose-dependent growth inhibitory effects were observed (Figure 1). The survival rates of 94.0%, 39.5%, 33.1%, and 23.0%, respectively, compared with that in non-Tan IIA-treated cells were detected after treatment with different concentrations of Tan IIA (0, 5, 10, 20, and 25 *μ*g/mL) for 24 hours. More than 90% of cells were killed with 25 *μ*g/mL of Tan IIA administration for 72 hours. The cytotoxic effects also became obvious as time passes when 10 *μ*g/mL of Tan IIA was added for 24, 48, and 72 hours; the survival rates were 39.5%, 27.7%, and 16.0%, respectively. Furthermore, nuclear morphological changes during apoptosis were observed using Hoechst staining assay (Figure 2(a)). After treatment of Tan IIA (0, 5, 10, and 20 *μ*g/mL), the apoptotic rates were 4.4%, 5.7%, 42.2%, and 93.9%, respectively, at 24 hours and 2.7%, 7.6%, 92.7%, and 98.6%, respectively, at 48 hours (Figure 2(b)). With higher dose and longer time period of administration, the apoptotic cells with shrunken and condensed nuclei became more prominent. Taken together, Tan IIA did induce oral KB cell death in a dose-dependent manner.

The article "Tanshinone IIA Induces Apoptosis in Human Oral Cancer KB Cells through a Mitochondria-Dependent Pathway" was retracted in 2017. Reasons: contaminated cell lines or tissues; unreliable results or conclusions.

### 3.2. Tanshinone IIA Arrested KB Cells in G_2_/M Phase

To evaluate the effect of Tan IIA on cell cycle progression, the cell cycle distribution was determined through flow cytometry analysis. After treatment with 10 *μ*g/mL of Tan IIA for 24 and 48 hours, there was an accumulation of cells in G_2_/M phase, while the cells in G_0_/G_1_ phase decreased compared with that in non-Tan IIA-treated cells (Figure 3). Moreover, the appearance of sub-G_1_ population indicated a proportion of apoptotic cell. The results suggested that Tan IIA-induced cell death might be involved in the induction of G_2_/M phase arrest and apoptosis.

### 3.3. Tanshinone IIA Induced the Loss of Mitochondrial Membrane Potential

The loss of mitochondrial membrane potential (ΔΨm) has been regarded as one of the early events in the apoptotic pathway, which can trigger the release of cytochrome c and other apoptogenic molecules after induction by various stimuli [20, 21]. To detect the change of the mitochondrial membrane potential, we used a mitochondria-specific and voltage-dependent dye, DiOC_6_, to stain the cells and then analyzed them through flow cytometry. As shown in Figure 4, KB cells treated with 10 *μ*g/mL of Tan IIA for 24 hours underwent the disruption of the mitochondrial membrane potential. Around 20% of the treated cells lost their mitochondrial membrane potential.

### 3.4. Tanshinone IIA Induced the Activation of Caspase-3, Caspase-9, and PARP

It is known that the apoptotic intrinsic pathway is initiated by intracellular stress, which dissipates transmembrane potential of mitochondrial membrane and results in the release of proapoptotic factors, including cytochrome c [20, 21]. The increased level of cytochrome c in the cytosol results in the initiation of caspase-9 and caspase-3 and the subsequent activation of PARP and induces the morphological changes of the dying cell [20–26]. In this signaling pathway, the specific PARP, a biochemical characteristic of apoptosis, mainly depends on the activation of caspase-3 [27]. In our study, western blot analysis was used to determine the effect of Tan IIA on caspase proteins and PARP. After exposure to different concentrations of Tan IIA (0, 5, 10, and 20 *μ*g/mL) for 24 hours, cellular proteins were lysed and immunoblotting was performed.  Figure 5 showed the activated subunits of caspase-9 with the decreased expression of procaspase-3 in Tan 20 group; a 116 kDa PARP was also cleaved to an 89 kDa fragment. The results suggested that Tan IIA-induced KB cell death was involved in the activation of caspase-3 and caspase-9 and the cleavage of PARP.

The article "Tanshinone IIA Induces Apoptosis in Human Oral Cancer KB Cells through a Mitochondria-Dependent Pathway" was retracted in 2017. Reasons: contaminated cell lines or tissues; unreliable results or conclusions.

## 4. Discussion

Tanshinone IIA (Tan IIA) is one major component of the dried root of* Salvia miltiorrhiza *Bunge. It acts as two faces in the biological and pharmacological effects. Some studies showed that Tan IIA is correlated with protection from cell death in cardiac myocytes and macrophage [14, 15]. However, others reported that Tan IIA has cytotoxic effects on several cancer cells [16–19]. The effects of Tan IIA on human oral cancer cells still remain unknown. The goal of this study is to investigate whether Tan IIA shows the anticancer effects on human oral cancer KB cells and to explore the possible underlying mechanism. Our findings indicate that Tan IIA inhibits cell proliferation, stops cell cycle progression, and induces apoptosis through the intrinsic mitochondrial pathway.

Apoptosis, one type of programmed cell death, is a well-defined self-suicide process counteracting tumor growth. Many chemotherapy drugs produce antitumor effects by triggering the apoptosis through a variety of molecular mechanisms [28]. As the natural phytochemicals have been increasingly employed as chemotherapy agents, we examined the cytotoxic effect of Tan IIA on KB cells and assessed the possible application of this ancient herbal medicine as a novel agent for treatment of oral cancer. In the present study, we demonstrated a naturally extracted Tan IIA inhibited the proliferation and viability of KB cancer cells in a dose-dependent manner using SRB colorimetric assay. More than 90% of cells were killed after administration with 25 *μ*g/mL of Tan IIA for 72 hours (Figure 1). Like studies mentioned above, Tan IIA did possess antiproliferative effects on human cancer cells. Furthermore, the cellular morphology was observed using Hoechst staining; those with shrunken and condensed fragmented chromosomes were identified as apoptotic cells (Figure 2(a)). Significant apoptosis developed when KB cells were treated with Tan 10 for 48 hours or Tan 20 for 24 and 48 hours (Figure 2(b)). Our results confirmed the involvement of apoptosis in response to Tan IIA in a dose-dependent manner.

Normal cell cycle progression is critical in regulating the cell proliferation and cell division. A dysregulation of the cell cycle that makes the cells undergo uncontrolled cell growth can result in the development of cancer. There are now more anticancer drugs that abrogate the cell cycle checkpoints and make the apoptosis develop [29, 30]. Thus, to target the errors of cell cycle regulation in cancer cells is considered a potential strategy for control of tumor growth. Previous studies showed that Tan IIA could arrest the nasopharyngeal carcinoma cell line (CNE-1) and human hepatocellular carcinoma cells (SMMC-7721) in G_0_/G_1_ phase, while other studies reported that human erythroleukemic cell line (K562) and HeLa cells were arrested in G_2_/M phase [16, 17, 31, 32]. When the cell cycle is arrested, there comes an opportunity for cells to undergo either a repairing mechanism or the apoptotic cascade. Prolonged mitotic arrest induced by microtubule-interfering agents such as taxol and vincristine had been proved to make cells enter apoptosis [33, 34]. Zhou et al. had found that Tan IIA arrested HeLa cells in mitosis through disrupting the mitotic spindle and triggered the apoptosis [17]. Our data indicated that Tan IIA caused the decrease of KB cells in G_0_/G_1_ phase, an accumulation in G_2_/M phase and an appearance in sub-G_1_ proportion (Figure 3). Thus, treatment of KB cells with Tan IIA induced G_2_/M phase arrest of cell cycle and the apoptosis indicating that Tan IIA might arrest cell cycle progression and lead to apoptosis.

The article "Tanshinone IIA Induces Apoptosis in Human Oral Cancer KB Cells through a Mitochondria-Dependent Pathway" was retracted in 2017. Reasons: contaminated cell lines or tissues; unreliable results or conclusions.

Apoptotic signaling processes tightly regulated by many antiapoptotic and proapoptotic molecules have been divided into extrinsic and intrinsic pathways. In the intrinsic mitochondrial apoptotic signaling,* Bcl-2 *has been identified as an apoptotic inhibitor and Bax protein inhibits the function of* bcl-2*. The apoptotic proteins, Bak and Bax, are key components that initiate mitochondrial dysfunction; an increased* Bax/Bcl-2 *ratio disrupts the mitochondrial membrane potential [35–37]. The loss of mitochondrial membrane potential is one of the characteristic biochemical changes in apoptosis. Yang et al. pointed out that Tan IIA caused the decrease in mitochondrial membrane potential of the EAhy926 human endothelial cells [19]. We observed that Tan IIA treatment led to the dissipation of mitochondrial membrane potential in partial KB cancer cells (Figure 4). Thus, a mitochondrial response was involved in the Tan IIA-induced apoptotic pathway of KB cancer cells. The loss of mitochondrial membrane potential results in the release of cytochrome c and other apoptogenic proteins from the mitochondria to cytosol. Consequently, the interaction between cytochrome c, apoptosis protease-activating factor 1, and ATP/dATP forms the apoptosome which activates caspase-9. The activation of caspase-9 causes the cleavage of caspase-3, a critical executioner of apoptosis. Subsequently the activated caspase-3 cleaves the substrates including PARP, ultimately leading to apoptosis [20–27]. Therefore, we evaluated the effect of Tan IIA on caspase proteins and PARP in KB cancer cells. Western blot analysis showed that Tan IIA treatment resulted in the activation of caspase-9, the triggering of caspase-3, and the cleavage of PARP in the KB cancer cells (Figure 5). Several studies also indicated that caspase-9, caspase-3, and PARP were associated with the Tan IIA-induced apoptosis on the cancer cell lines [16, 17, 19]. Taken together, Tan IIA treatment led to the initiation of the intrinsic mitochondrial pathway and the activation of downstream caspase-3 in apoptosis of human oral cancer KB cells.

The article "Tanshinone IIA Induces Apoptosis in Human Oral Cancer KB Cells through a Mitochondria-Dependent Pathway" was retracted in 2017. Reasons: contaminated cell lines or tissues; unreliable results or conclusions.

## 5. Conclusion

In conclusion, our study shows that Tan IIA suppresses the cell growth, arrests cells in G_2_/M phase, and induces the apoptotic cell death of human oral cancer KB cells. In addition, we find that Tan IIA induces the apoptosis of KB cells through mitochondrial-dependent pathway in which the loss of mitochondrial membrane potential and the activation of caspase-9 and caspase-3 are involved, though other routes may be associated with the apoptotic events and need further investigation. Data obtained from our study indicate that Tan IIA could be a potential anticancer agent for oral cancer.

## Figures and Tables

**Figure 1:** Effect of Tan IIA on KB cell proliferation. KB cells were treated with different concentrations of Tan IIA (0, 5, 10, 20, and 25 *μ*g/mL) for 24, 48, and 72 hours. The cell cytotoxicity and viability were detected by SRB colorimetric assay. Values are the mean ± SD of 3 independent experiments. ∗ indicates *P* < 0.05.

**Figure 2:** Assessment of nuclear morphological changes of KB cells exposed to Tan IIA. KB cells were treated with various contractions of Tan IIA (0, 5, 10, and 20 *μ*g/mL) for different time periods. (a) After 24 hours, cells stained with Hoechst and exhibiting shrunken, condensed nuclei with fragmented chromosomes under fluorescent microscope were identified as apoptotic cells. (b) Apoptotic rates were calculated. The points are the mean ± SD of 2 independent experiments. ∗ indicates *P* < 0.05.

**Figure 3:** Effect of Tan IIA on cell cycle of KB cells. KB cells were treated with Tan IIA (0, 5, and 10 *μ*g/mL) for 24 and 48 hours. Harvested cells were stained by propidium iodide and analyzed by flow cytometry. Values are the mean ± SD of 4 independent experiments. ∗ indicates *P* < 0.05.

**Figure 4:** Influence of Tan IIA on the mitochondrial membrane potential (ΔΨm) of KB cells. KB cells were treated with Tan IIA (0, 5, and 10 *μ*g/mL) for 24 hours. After DiOC_6_ staining, the changes of the mitochondrial membrane potential were measured using flow cytometry. Values are the mean ± SD of 4 independent experiments. ∗ indicates *P* < 0.05.

The article "Tanshinone IIA Induces Apoptosis in Human Oral Cancer KB Cells through a Mitochondria-Dependent Pathway" was retracted in 2017. Reasons: contaminated cell lines or tissues; unreliable results or conclusions.

**Figure 5:** Effect of Tan IIA on caspase proteins and PARP of KB cells. Lysates of the KB cells treated with Tan IIA (0, 5, 10, and 20 *μ*g/mL) for 24 hours were subjected to an immunoblot analysis with antibodies against caspase-3, caspase-9, and PARP. *β*-actin was served as the loading control.
